# Multiset Canonical Correlations Analysis of Bidimensional Intrinsic Mode Functions for Automatic Target Recognition of SAR Images

**DOI:** 10.1155/2021/4392702

**Published:** 2021-08-25

**Authors:** Yong Ding

**Affiliations:** Zhejiang Institute of Economics and Trade, Hangzhou 310018, China

## Abstract

A novel feature generation algorithm for the synthetic aperture radar image is designed in this study for automatic target recognition. As an adaptive 2D signal processing technique, bidimensional empirical mode decomposition is employed to generate multiscale bidimensional intrinsic mode functions from the original synthetic aperture radar images, which could better capture the broad spectral information and details of the target. And, the combination of the original image and decomposed bidimensional intrinsic mode functions could promisingly provide more discriminative information for correct target recognition. To reduce the high dimension of the original image as well as bidimensional intrinsic mode functions, multiset canonical correlations analysis is adopted to fuse them as a unified feature vector. The resultant feature vector highly reduces the high dimension while containing the inner correlations between the original image and decomposed bidimensional intrinsic mode functions, which could help improve the classification accuracy and efficiency. In the classification stage, the support vector machine is taken as the basic classifier to determine the target label of the test sample. In the experiments, the 10-class targets in the moving and stationary target acquisition and recognition dataset are classified to investigate the performance of the proposed method. Several operating conditions and reference methods are setup for comprehensive evaluation.

## 1. Introduction

With the fast progress in SAR technologies, the massive radar measurements can hardly be interpreted by mere human intervention. In this context, the ATR system is developed, which comprises an integrated gallery of algorithms handling different tasks [1–3]. In the SAIP system [2], the famous three-stage processors were designed for SAR ATR, i.e., detection, discrimination, and classification. The detector locates the ROI by searching through a large-scene image, which may cover several square kilometers of ground. Afterwards, the discriminator operates the preliminary classification to distinguish the man-made objects and natural clutters. And, those ROIs assumed to be natural clutters are discarded. The classification procedure is performed finally to obtain target labels. As the core index of a SAR ATR system, the recognition performance is directly related to the used classification scheme. In the past decades, a rich collection of available feature extraction algorithms and classifiers were used for SAR ATR owing to the progress in modern pattern recognition techniques. The features are first extracted from the original SAR images before the classification, which are used to describe the target characteristics. The hand-crafted features for SAR ATR are obtained via inheriting the optical image processing techniques as well as considering the unique properties of SAR images, such as geometrical, transformation, and scattering features. Geometrical features are classical ones, which have been adopted in optical image processing for a long time [4–9]. Also, they are used to describe the geometric properties of SAR targets such as sizes and shapes. In [4], the descriptors of target outline, i.e., EFS, were extracted for classification. Amoon and Clemente generated the moments' features, i.e., Zernike [5] and Krawtchouk [6] moments, respectively, from the binary target regions segmented from SAR images, which were afterwards classified for target recognition. Ding et al. directly matched two binary target regions from the test sample and corresponding templates for SAR target recognition [7]. The transformation features are constructed via mathematical projection or signal processing to depict the intensity distribution or spectral properties of the original images [10–17]. The manifold learning algorithms are applied to SAR image feature extraction including linear and nonlinear ones. Typical examples of linear methods are LDA [10], PCA [10, 11], and NMF [12]. To handle the possible nonlinearity embedded in the data, some nonlinear manifold algorithms are also developed for feature extraction [13, 14]. Several signal processing techniques are extended to image processing such as wavelet analysis [15] and monogenic signal [16, 17]. In [16, 17], the researchers introduced monogenic signal analysis to feature extraction of SAR images, which is demonstrated highly effective for SAR ATR. Unlike the optical imaging mechanism, SAR images reflect the electromagnetic scatterings of the target [18]. In this sense, the scattering features, e.g., attributed scattering centers, are also sufficiently descriptive to distinguish different kinds of targets, which provide locally relevant descriptions of the target structures. The effectiveness of attributed scattering centers was experimentally investigated in some previous works [19–21]. The classifiers were also greatly enriched over the past decades. The SAIP system employed the template matching as the baseline classifier. In [22], Zhao and Principe introduced SVM into SAR ATR, which became one the most popular classifier in this field [4, 5, 23, 24]. The development in compressive sensing theory produced a robust classifier called SRC [25–28], which was used by Thiagarajan et al. to handle SAR ATR issues. Other classifiers such as AdaBoost [29], discriminative graphic model [30], modified polar mapping classifier [31], and HMM [9] were also investigated in the field of SAR ATR. As the deep learning methodology is getting mature, the deep classifiers for image interpretation, e.g., CNN [32–37], were validated highly effective for SAR ATR. However, the performance of CNN is highly dependable on the amount of available training samples. As a remedy, some CNN-based methods sought performance enhancement via proper data augmentations [34, 35].

In this paper, we propose a new way of generating discriminative features for SAR ATR via BEMD [38] and MCCA [39]. EMD adaptively decomposes 1D nonstationary signals, which was proposed by Huang et al. [40]. With no prior assumptions on the data properties, e.g., linearity or stationarity, EMD could keep its effectiveness and robustness under different conditions. As a natural extension, BEMD is capable of analyzing 2D signals, e.g., images, to learn more details. Via the sifting process, the generated BIMFs could provide complementary information for the original image, thus beneficial for image interpretation such as image denoising and image fusion [41–46]. Owing to these merits, we introduce BEMD to SAR feature extraction. In this way, much broader spectral properties of the original SAR images can be captured by the BIMFs for the following classification tasks. The BIMFs are also images with the same sizes of the original one. As a result, they significantly increase the computational burden of classification. As a feasible solution, some feature extraction algorithms could be used to reduce their dimensions independently, such as the down-sampling strategy for the multiscale monogenic components used in [16]. However, such strategies neglect the inner correlations between the original image and BIMFs, which are also beneficial to distinguish different classes. As a remedy, this study employs MCCA to fuse the original SAR image and decomposed BIMFs as a unified feature vector. CCA provides a statistical way to analyze the relationship between two random variables and find the best projection matrices to keep their correlations [47]. MCCA extends CCA to multiple random variables [48–52]. The resulted feature vector could significantly reduce the high dimension of the original image and BIMFs, while maintaining their inner correlations; thus, both the efficiency and effectiveness of the following classification can be promisingly enhanced. To perform the classification task, SVM is adopted as the classifier. SVM is one of the most popular classifiers used in SAR ATR. In the previous literature, SVM was employed to classify various kinds of features, e.g., target outline descriptors, region moments, and PCA feature vectors, with good performance. Therefore, we use SVM to classify the fused feature vector via MCCA to determine the target label of the test sample. The main contribution of this study is that a novel feature extraction method is proposed via the combination of BEMD and MCCA. The resulted features can maintain the discrimination in the original image and its BIMFs with a significantly low dimension. Therefore, the highly discriminative features can effectively improve the classification performance.

The remaining sections of this paper are organized as follows.  Section 2 introduces the main methodology of the proposed method including BEMD, MCCA, and SVM. In Section 3, experimental investigations are conducted on the MSTAR dataset to evaluate the performance of the proposed method.  Section 4 discusses the experimental results, and Section 5 draws some conclusions to summarize this paper. The acronyms used throughout the whole paper are summarized in Table 1.

## 2. Methodologies of the Proposed Method

### 2.1. BEMD

Different from stationary signals, nonstationary ones vary along with time thus much difficult to be reliably analyzed. Proposed by Huang et al. [41], EMD provides an adaptive way to decompose 1D signals. Unlike traditional signal decomposition algorithms, e.g., Fourier transform and wavelet analysis, EMD does not design predetermined basis functions but adaptively conducts the decomposition according to the properties of the data.

The IMFs are decomposed from EMD, which could be used to better analyze the time-frequency properties of the original image. Owing to its adaptivity and stability, EMD has been successfully applied to process different kinds of signals including biological, medical, and astronomy ones. Given an original signal as *f*(*t*), the decomposition process of EMD (often called “sifting”) is formulated as follows:

(1) $$\begin{array}{c} f\left(t\right)=\sum_{k=1}^{K}J_{k}\left(t\right)+r_{K}\left(t\right), \end{array}$$

where *J*_*k*_(*t*), *k*=1,2,…, *K*, represents the IMFs and *r*_*K*_ denotes the residue.

To handle 2D signals such as images, Nunes et al. generalized the original EMD to BEMD. Similarly, via BEMD, an image is decomposed to several BIMFs to provide more detailed descriptions for it. According to Nunes et al. [38], for a given image *I*(*i*, *j*) with the sizes of *M* × *N*, the sifting process of BEMD is summarized as the following steps:

*Step* 1. Identify the locations of the local extrema (including the maxima and minima) in *I*(*i*, *j*).
*Step* 2. Generate the envelopes according to the maxima and minima point sets via 2D interpolation, respectively. Afterwards, the local mean *m* is computed as the average of the upper (from the maxima points) and lower (from the minima points) envelopes.
*Step* 3. Subtract the local mean from the original image to get a proto-BIMF as *r*=*I* − *m*. If *r* is judged to be a BIMF, go to *Step* 4. On the contrary, it is used as the input to repeat *Steps* 1 and 2 until the latest proto-BIMF becomes a BIMF.
EMD sifting was iterated based on the Cauchy standard deviation criterion designed by Huang et al. For the case of BEMD, the criterion is updated as follows:
  (2) $$\begin{array}{c} SD=\sum_{i=1}^{M}\sum_{j=1}^{N}\frac{{\left(r_{k}\left(i,j\right)-r_{k-1}\left(i,j\right)\right)}^{2}}{r_{k-1}^{2}\left(i,j\right)}, \end{array}$$
where *r*_*k*_(*i*, *j*) is the output in the *k*th iteration and *r*_*k*−1_(*i*, *j*) is the result from the (*k* − 1)th iteration. Based on the calculated SD value, the sifting process is judged to continue or stop. When the SD is larger than a predefined threshold *ε*, the sifting process continues by repeating *Steps* 1 to 3 with *r*_*k*_(*i*, *j*) as the input. On the contrary, *r*_*k*_(*i*, *j*) is judged to be a BIMF *d*_*k*_(*i*, *j*), which is output. According to the analysis in [35], we set *ε*=0.12 in this paper as a suitable choice of the threshold.
*Step* 4. Take the proto-BIMF *r* as the input and repeat *Steps* 1 to 3 to obtain the next BIMF until the process can be looped further.

After the sifting process, the original image can be represented as the combination of the BIMFs as follows:

(3) $$\begin{array}{c} I\left(i,j\right)=\sum_{k=1}^{K}{\text{d}}_{k}\left(i,j\right)+r_{K}\left(i,j\right). \end{array}$$

In equation (3), *d*_*k*_(*i*, *j*) denotes the *k*th BIMF and *r*_*K*_(*i*, *j*) represents the final residual. Among all the BIMFs, *d*_1_ describes the highest frequency of *I* and *r*_*K*_(*i*, *j*) represents the lowest frequential component. Therefore, the multiscale BIMFs could provide more comprehensive descriptions of the spectral properties of the original image. In addition, some details can be better embodied in the BIMFs, which cannot be remarkably reflected in the original image. Therefore, by proper use of the BIMFs, more information of the original image can be exploited for the interpretation tasks such as image denoising, image fusion, and image classification.

The advantages of BEMD inspires us to apply it to feature extraction of the SAR image for target recognition.  Figure 1 intuitively displays the effectiveness of BEMD on the SAR target image chips from the MSTAR dataset, in which the first three BIMFs are shown. It can be observed that some details (e.g., the dominant scattering centers) in the original images can be better reflected in the first two BIMFs. In the third BIMF, the target related descriptions become blurry. As a result, it provides very limited discrimination for target recognition. Accordingly, only the first two BIMFs are used for target recognition in the following.

### 2.2. MCCA

CCA provides a statistical way to identify the association between two sets of random variables. As a generalization of CCA, MCCA is capable of analyzing the relationships among more sets of variables [48–52]. Assume that there are *n* random vectors *X*_*i*_ ∈ *R*^*pi*^(*i*=1,2,…, *n*) and each of them is centralized to have *E*(*X*_*i*_)=0, in which *pi* corresponds to the dimension of *X*_*i*_. MCCA aims to find the linear combinations *U*=[*U*_1_, *U*_2_,…, *U*_*n*_] of *X*^*T*^=[*X*_1_^*T*^, *X*_2_^*T*^,…, *X*_*n*_^*T*^] given by

(4) $$\begin{array}{c} U_{1}=\alpha_{1}^{T}X_{1},\text{Var}\left\{U_{1}\right\}=\alpha_{1}^{T}S_{11}\alpha_{1},\\ U_{1}=\alpha_{1}^{T}X_{1},\text{Var}\left\{U_{1}\right\}=\alpha_{1}^{T}S_{11}\alpha_{1},\\ \begin{array}{ccc} \; & \vdots & \; \end{array}\;\begin{array}{ccc} & \vdots & \; \end{array}\;\begin{array}{ccc} \; & & \vdots \end{array}\\ U_{n}=\alpha_{n}^{T}X_{n},\text{Var}\left\{U_{n}\right\}=\alpha_{n}^{T}S_{nn}\alpha_{n}, \end{array}$$

with the dispersion matrix as follows:

(5) $$\begin{array}{c} \Sigma_{U}=\left(\begin{array}{ccc} \alpha_{1}^{T}S_{11}\alpha_{1} & \ldots & \alpha_{1}^{T}S_{1n}\alpha_{n}\\ \vdots & \ddots & \vdots \\ \alpha_{n}^{T}S_{n1}\alpha_{n} & \ldots & \alpha_{n}^{T}S_{nn}\alpha_{n} \end{array}\right), \end{array}$$

where *S*_*ij*_ represents the covariance matrix between *X*_*i*_(*i*=1,2,…, *n*) and *X*_*j*_(*j*=1,2,…, *n*) and *S*_*ii*_ denotes the covariance matrix of vector *X*_*i*_, and the vector *α*_*i*_ ∈ *R*^*pi*^. MCCA searches for the projection vectors *α*_1_, *α*_2_,…, *α*_*n*_, which maximize the correlations between the canonical variables *U*_1_, *U*_2_,…, *U*_*n*_. A measure to evaluated their correlations can be formulated in terms of the covariance matrices. Then, the measure of Σ_*U*_ can be optimized by imposing special criteria with some constraints. One of the well-known criteria called “SUMCOR” is exhibited in the following equation:

(6) $$\begin{array}{c} \left(\alpha_{1},\alpha_{2},\ldots ,\alpha_{n}\right)=\underset{\alpha_{1},\alpha_{2},\ldots ,\alpha_{n}}{\max}\sum_{i=1}^{n}\sum_{j=1}^{n}\alpha_{i}^{T}S_{ij}\alpha_{j},\\ \text{s.t.}\;\sum_{i=1}^{n}\alpha_{i}^{T}S_{ii}\alpha_{i}=1. \end{array}$$

To solve the problem in equation (6), the Lagrange multiplier technique can be used. It can be reformulated as equation (7) as solving the generalized eigenvalue problem:

(7) $$\begin{array}{c} \left(\begin{array}{ccc} S_{11} & \ldots & S_{1n}\\ \vdots & \ddots & \vdots \\ S_{n1} & \ldots & S_{nn} \end{array}\right)\left(\begin{array}{c} \alpha_{1}\\ \vdots \\ \alpha_{n} \end{array}\right)=\lambda \left(\begin{array}{ccc} S_{11} & \ldots & 0\\ \vdots & \ddots & \vdots \\ 0 & \ldots & S_{nn} \end{array}\right)\left(\begin{array}{c} \alpha_{1}\\ \vdots \\ \alpha_{n} \end{array}\right). \end{array}$$

The optimal projections vectors for *X*_*i*_ are calculated as the conjugate eigenvectors *α*_*i*1_, *α*_*i*2_,…, *α*_*id*_ corresponding to the first *d*=min(*p*1, *p*2,…, *pn*) eigenvalues *λ*_*i*1_ ≥ *λ*_*i*2_ ≥ ⋯≥*λ*_*id*_ in equation (7). Afterwards, the multiset canonical correlation vectors can be obtained as the following equation:

(8) $$\begin{array}{c} U_{i}=\left(\alpha_{i1}^{T}X_{i},\alpha_{i2}^{T}X_{i},\ldots ,\alpha_{id}^{T}X_{i}\right),\\ ={\left(\alpha_{i1},\alpha_{i2},\ldots ,\alpha_{id}\right)}^{T}X_{i}=W_{i}^{T}X_{i}, \end{array}$$

where *W*_*i*_=[*α*_*i*1_, *α*_*i*2_,…,*α*_*i*  *d*_]_*pi*×*d*_(*i*=1,2,…, *n*) represents the projection matrix for each set of the random variables.

As discussed above, MCCA is capable of exploiting the within-set and between-set correlations among multiple vectors. Therefore, it can be used to fuse multiple random variables to reduce the redundancy, while maintaining the correlations. In this work, the serial fusion strategy (Peng et al. [48]) is adopted as the following equation:

(9) $$\begin{array}{c} Z=W_{1}^{T}X_{1}+W_{2}^{T}X_{2}+\cdots +W_{n}^{T}X_{n}, \end{array}$$

where *Z* denotes the fused feature vector.

### 2.3. Target Recognition via SVM

SVM is chosen as the classifier to classify the generated features for target recognition. Since the first proposal by Vapnik et al. in 1995, SVM has been widely used in the pattern recognition problems. In 2001, it is introduced into SAR ATR by Zhao and Principe [22]. After then, SVM became one of the most popular classifiers in SAR ATR. According to the structural risk minimization principle, the preliminary SVM finds a hyperplane to separate patterns from two different classes. The decision function for a test sample *x* in SVM can be formulated as follows:

(10) $$\begin{array}{c} f\left(x\right)=\sum_{i=1}^{M}w_{i}y_{i}K\left(x_{i},x\right)+b\text{,}\;\alpha_{i}\geq 0,\forall i. \end{array}$$

In equation (10), *x*_*i*_(*i*=1,…, *M*) denotes a support vector from the training samples and *y*_*i*_=±1 is its corresponding label. *w*_*i*_(*i*=1,…, *M*) and *b* (bias) are the parameters estimated during the training. *K*(*·*) represents the kernel function. With different choices of kernel functions, the trained SVM can handle different kinds of classification problems including linear and nonlinear ones. The polynomial kernel and RBF kernel are two typical kernel functions in SVM.

Researchers generalized the two-class SVM to multiclass one via the one-versus-one or one-versus-rest strategies. In this way, SVM can be directly used to classify many types of targets simultaneously. The famous LIBSVM [53] is an excellent toolbox to employ SVM for different usages, which is also used in this work. The multiclass SVM with the RBF kernel is adopted to perform the classification tasks based on the generated features.

The novel feature vectors generated by BEMD and MCCA are classified by SVM, as shown in Figure 2. Considering that the original image and BIMFs are all 2D matrices, they are reshaped as 1D vectors. Afterwards, MCCA is employed to fuse them as a unified feature vector. In detail, the following steps are implemented to perform the target recognition task.

  Step 1: BEMD is used to extract the multiscale BIMFs from the training samples
  Step 2: the first two BIMFs and original image are taken as random variables to calculate the projection matrices using MCCA
  Step 3: each of the training samples and its corresponding BIMFs are fused based on the projection matrices from Step 2 to build a new training set
  Step 4: the fused feature vector of the test sample is obtained using BEMD and MCCA in the same way with the training samples
  Step 5: the feature vector of the test sample is classified by SVM to determine the target label

## 3. Experiments

### 3.1. Dataset and Methods for Comparison

The MSTAR dataset is employed for experimental evaluation in this study, which is widely used to develop and test SAR ATR algorithms. There are 10 representative ground targets contained in the dataset, whose optical appearances are displayed as Figure 3. SAR images of these targets are acquired by X-band sensors with the resolution of 0.3 m × 0.3 m. The aspect angles of each target cover full 0°∼360° at different depression angles, e.g., 15°, 17°, 30°, and 45°. In addition, some targets (e.g., BMP2 and T72) have several different configurations with some structural modifications.

As a necessary part of validating the performance of the proposed method, some baseline algorithms, which are widely used in SAR ATR, are compared. Their implementation details are itemed as follows.

- SVM + PCA [11]: the 80-dimension projection features extracted by PCA are used to represent the original SAR images. SVM is used as the classifier in the classification stage.
- SVM + Zernike [5]: the Zernike moments of the binary target region are used as the basic features. SVM is used as the classifier in the classification stage.
- SVM + EFS [4]: the descriptors of target outline, i.e., EFS, are used as the basic features. SVM is used as the classifier in the classification stage.
- SRC [25]: random projection is adopted to reduce SAR images to 1024-dimension feature vectors. SVM is used as the classifier in the classification stage.
- A-ConvNet [32]: the raw image intensities are directly used to represent the original images. The all-convolutional networks are taken as the classifier.
- ESENet [33]: the ESENet is employed for SAR ATR.
- JSRDeep [36]: the CNN is developed for feature learning to generate multilayer feature maps. Afterwards, the joint sparse representation is employed to classify the deep feature vectors.

Specifically, this paper employs the LIBSVM package developed by Lin et al. to perform the multiclass SVM classification. The SparseLab package [54] is employed to solve the sparse representation problem in SRC. And, CNN is trained on the TensorFlow platform.

The following experiments are conducted under both the SOC and EOCs to fully evaluate the effectiveness of the proposed method. At last, the performance of the proposed method and baseline algorithms are compared under different conditions to reach more intuitive evaluations on the proposed method.

### 3.2. Results under SOC

The proposed method is first investigated under SOC, which can be regarded as a preliminary verification.  Table 2 shows the training and test samples from the 10 classes under SOC. Images at 17° depression angle are trained for the classification of 15°-depression-angle test samples. Specifically, the test images of BMP2 and T72 contain two more configurations (i.e., SNs) than their training sets, respectively. The confusion matrix is used to display the classification results by the proposed method as Figure 4, in which the *X* and *Y* coordinates represent the predicted and actual labels, respectively. It shows that each class can be classified with a recognition rate over 97.5%. And, the overall recognition rate of the 10 targets is averaged to be 99.03%. Because of the existing configuration differences between the training and test sets, BMP2 and T72 get the lowest two recognition rates among all the targets. According to the reported results, the high performance of the proposed method under SOC is quantitively validated. The BIMFs generated by BEMD are discriminative features, which could maintain the original target characteristics. Furthermore, MCCA combines the original image and its multiscale BIMFs as a unified feature vector, while keeping the inner discrimination. Finally, as a high-performance classification scheme, SVM makes decisions on the target labels based on the fused features. All these factors contribute to the excellent performance of the proposed method under SOC.

### 3.3. Recognition under EOC

EOCs are common situations in SAR ATR. As illustrated in Table 2, the same target may have different configurations. Moreover, due to the variations of backgrounds and sensors, other EOCs such as depression angle variance and noise corruption are also severe obstacles to the smooth implementation of SAR ATR systems. Consequently, in this part, three typical EOCs are setup to test the robustness of the proposed method. The first EOC is configuration variance and the training and test samples are displayed in Table 3. For BMP2 and T72, their test samples are from totally different SNs with the training ones. In addition, BDRM2 and BTR70 are used as two confuser targets in the training set, which further increases the difficulty of correct classification. The training and test samples for the second EOC are presented in Table 4 including SAR images of four targets (2S1, BDRM2, ZSU23/4, and T72 (SN_A64)) from different depression angles. Samples at 17° depression angle are trained for the classification of test samples at 30° and 45° depression angles, respectively. The relatively large depression angle variances between the training and test samples decrease their similarities in SAR images [55], as shown in Figure 5. The third EOC is noted as “noise corruption.” According to ideas in [16, 32], the noisy samples are obtained by adding random noises into the original test images in Table 2. In detail, a certain percentage of pixels in the original SAR images are replaced by impulses, i.e., pixels with large intensities.  Figure 6 illustrates some noisy samples at different noise levels.

Based on the aforementioned EOC experimental setups, the robustness of the proposed method is tested.  Table 5 displays the classification results of the proposed method under EOC-1. The test configurations of BMP2 and T72 can all be classified with recognition rates over 96%. And, the overall recognition rate is 98.08%. As shown in Figure 1, the multiscale BIMFs can better reflect the detailed information in the original SAR image. The local variations caused by configuration variances can be possibly embodied in the BIMFs. Therefore, the combination of the original image and BIMFs can help improve the classification accuracy under configuration variance. The classification results of the proposed method under EOC-2 are presented in Table 6. The average recognition rates at 30° and 45° depression angles achieved by the proposed method are 98.18% and 73.43%, respectively. The great decrease in recognition rate at 45° depression angle is probably caused by the low similarities between the training and test samples, which can be observed in Figure 5.  Table 7 lists the average recognition rates at different noise levels, which shows the sensitivity of the recognition performance to random noise corruption. At 20% noise level, the overall recognition rate jumps to 62.12%, which is significantly lower than that on the original test samples. As a summary, the proposed method is investigated under both SOC and three typical EOCs. Compared with EOCs, the performance under SOC is much better because the test samples are much more similar with the training ones. In each EOC, the classification accuracy is closely related to the deterioration degree, which can be directly seen from the results in EOC-2 and EOC-3.

### 3.4. Performance Comparison with Baseline Algorithms

In this part, the proposed method is evaluated against the baseline algorithms under different operating conditions.  Table 8 compares the performance of all the methods under SOC and EOC-1. The proposed method outperforms the others under both situations. In contrast to other three SVM-based methods, the proposed method achieves 2.11%, 2.89%, and 2.61% increments in the recognition rate over PCA, Zernike, and EFS features under SOC. And, the increments change to 3.21%, 2.94%, and 2.88% under EOC-1. The better performance achieved by the proposed method verifies the superior effectiveness of the features used in the classification stage. Therefore, the generated features via combination of BIMFs and MCCA are more discriminative than the projection features extracted by PCA, region features (e.g., Zernike moments), and target outlines (e.g., EFS descriptors).  Figure 7 simultaneously compares the recognition rates of all the methods at different depression angles. With a similar trend occurred in the proposed method, the baseline algorithms all decrease sharply when the depression angle switches from 30° to 45°. At each depression angle, the proposed method gains the highest accuracy mainly because the generated features can better reflect the local variations caused by depression angle variance. Especially at 45° depression angle, the predominance of our approach becomes much more obvious and the least increment in the recognition rate is over 3.41% in comparison with the baseline algorithms. The performance of different methods under random noise corruptions is shown in Figure 8. Although decreasing with the aggravation of the noise level, the recognition rates of the proposed method keep higher than those of the baseline algorithms. So, the generated features are more robust than the other features according to the experimental results. The Zernike and EFS features perform relatively better among the baseline algorithms because the two types of features are extracted based on the binary target region, which keeps more robust than the intensity distributions under random noises. For the CNN-based methods, they are relatively more vulnerable to random noise corruption than the remaining ones. According to the deep learning classification scheme, the performance is highly attributed to the coverage of the training set. Under high levels of random noises, the operating conditions of the test samples cannot be covered by the original training samples. As a result, the classification accuracy decreases sharply. According to the results of performance comparison, the superiority of the proposed method under both SOC and EOCs is validated. And, the main reasonability of the good performance lies in the high discriminability of the generated features via the combination of BIMFs and MCCA.

## 4. Discussions

Some discussions are made in this section to further explain the experimental results on the MSTAR dataset, which quantitively verified the superior performance of the proposed method. The reasonability and feasibility of the results can be discussed from following aspects.

1. The high discrimination capability of the generated feature via BEMD and MCCA: the multiscale BIMFs extracted by BEMD can capture broader spectral information of SAR images. As displayed in Figure 1, more details of the target can be reflected in the BIMFs than the original image. Therefore, by combining the original image and decomposed BIMFs, more discriminative information is available for the following classification. As a statistical information fusion algorithm, MCCA could fuse the original image and decomposed BIMFs as a unified feature vector with a low dimension, while maintaining the inner correlations among them. Therefore, the generated features via BEMD and MCCA are discriminative for SAR ATR.
2. The effectiveness and robustness of SVM for target classification: SVM is a classical and popular classifier in pattern recognition applications. Also, it has been widely employed in SAR ATR with good extension capability to different types of features. Therefore, it is a suitable classifier for the generated features in our study.
3. Experimental results under SOC: SOC refers to the operating condition, under which the test and training samples keep high similarities. Therefore, it is predictable that the recognition algorithms could perform well under SOC. The proposed method attains a recognition rate of 99.12% under SOC, higher than those of the baseline algorithms. The results validate the superiority of the proposed method.
4. Experimental results under EOCs: EOC refers to the operating condition, under which the test and training samples have notable differences. As a result, it is a much harder classification task than SOC problems. Three typical EOCs (configuration variance, depression angle variance, and random noise corruption) are setup to comprehensively examine the robustness of the proposed. Compared with the baseline algorithms, the proposed one achieves better performance under different types of EOCs.

## 5. Conclusions

This paper proposes a feature generation method for SAR images for target recognition. The multiscale BIMFs are first obtained from the original image by BEMD, which provide more detail information of the target. To enhance the classification accuracy and efficiency in the following stage, MCCA is employed to combine the original image and decomposed BIMFs as a unified feature vector. Because MCCA constructs the projection matrices by considering the relationship between different components, the resulted feature vector actually reflects the inner correlations of the original image and decomposed BIMFs. SVM is adopted as the classifier to classify the generated feature vector. According to the experimental investigations on the MSTAR dataset under different kinds of operating conditions, several conclusions could be reached as follows: (1) BEMD could extract discriminative representations, i.e., BIMFs, from SAR images. The multiscale BIMFs help capture broader spectral information and reflect more details of the original image. So, they can complement the original image to provide more discrimination to improve the recognition performance. (2) MCCA is an effective method to combine the original SAR image and decomposed BIMFs. The generated low-dimensional feature vector contains the inner correlations between different components. (3) As an overall evaluation, the proposed achieves better performance than some baseline SAR ATR methods. Especially, the robustness of the proposed method under several typical EOCs including configuration variance, depression angle variance, and random noise corruption is much more superior. In the future, in order to better handle the uncertainties caused by EOCs, feature extraction, etc., the fuzzy theory [56, 57] may be a potential way to further improve the recognition performance.

## Figures and Tables

**Figure 1:** Feature extraction of the SAR image by BEMD.

**Figure 2:** Implementation of target recognition based on the features generated by BEMD and MCCA.

**Figure 3:** Optical appearances of the 10 targets in MSTAR dataset. (a) BMP2, (b) BTR70, (c) T72, (d) T62, (e) BRDM2, (f) BTR60, (g) ZSU23/4, (h) D7, (i) ZIL131, and (j) 2S1.

**Figure 4:** Classification results of the proposed method under SOC.

**Figure 5:** Comparison of SAR images from different depression angles. (a) 17°. (b) 30°. (c) 45°.

**Figure 6:** Exemplar images with different levels of random noises under EOC-3: noise corruption. (a) 0%; (b) 5%; (c) 10%; (d) 15%; (e) 20%.

**Figure 7:** Comparison under EOC-2.

**Figure 8:** Comparison under EOC-3.

**Table 1:** The acronyms used in this paper.

Full name	Acronyms
Synthetic aperture radar	SAR
Automatic target recognition	ATR
Semiautomated image intelligence processing	SAIP
Region of interests	ROI
Elliptical Fourier series	EFS
Linear discriminant analysis	LDA
Principal component analysis	PCA
Nonnegative matrix factorization	NMF
Support vector machine	SVM
Sparse representation-based classification	SRC
Adaptive boosting	AdaBoost
Hidden Markov model	HMM
Convolutional neural networks	CNN
Bidimensional empirical mode decomposition	BEMD
Multiset canonical correlations analysis	MCCA
Empirical mode decomposition	EMD
Canonical correlations analysis	CCA
Bidimensional intrinsic mode function	BIMF
Intrinsic mode function	IMF
Moving and stationary target acquisition and recognition	MSTAR
Radial basis function	RBF
Standard operating condition	SOC
Extended operating condition	EOC
Serial number	SN

**Table 2:** Training and test samples under SOC.

	BMP2	BTR70	T72	T62	BDRM2	BTR60	ZSU23/4	D7	ZIL131	2S1
Training	233 (SN_9563)	233	232 (SN_132)	299	298	256	299	299	299	299

Test	195 (SN_9563)	196	196 (SN_132)	273	274	195	274	274	274	274
	196 (SN_9566)		195 (SN_812)							
	196 (SN_C21)		191 (SN_S7)							

**Table 3:** Training and test samples for EOC-1: configuration variance.

	BMP2	BDRM2	BTR70	T72
Training (17°)	233 (SN_9563)	298	233	232 (SN_132)

Test (15°, 17°)	428 (SN_9566)	0	0	426 (SN_812)
				429 (SN_C21)
				573 (SN_A04)
				573 (SN_A05)
				573 (SN_A07)

**Table 4:** Training and test samples for EOC-2: depression angle variance.

	Depr.	2S1	BDRM2	ZSU23/4	T72 (SN_A64)
Training	17°	299	298	299	299

Test	30°	288	287	288	288
	45°	303	303	303	303

**Table 5:** Results of the proposed method under EOC-1.

Class	Configuration	BMP2	BRDM2	BTR70	T72	Recognition rate (%)
BMP2	SN_9566	420	3	2	3	98.13
	SN_C21	424	1	1	3	98.83

T72	SN_812	1	3	3	417	98.36
	SN_A04	5	1	3	564	98.43
	SN_A05	7	4	2	560	97.73
	SN_A07	9	1	4	559	97.56
	SN_A10	8	3	3	553	97.53

Overall						98.08

**Table 6:** Results of the proposed method under EOC-2.

Depr.	Actual	Predicted				Recognition rate (%)	Overall (%)
		2S1	BRDM2	ZSU23/4	T72		
30°	2S1	283	1	3	1	98.26	98.18
	BDRM2	2	284	0	1	98.95	
	ZSU23/4	4	1	281	2	97.57	
	T72	2	4	0	282	97.92	

45°	2S1	216	47	23	17	71.29	73.43
	BDRM2	29	234	21	19	77.23	
	ZSU23/4	18	43	213	29	70.30	
	T72	20	25	31	227	74.92	

**Table 7:** Results of the proposed method under EOC-3.

Noise level (%)	5	10	15	20
Recognition rate (%)	93.54	86.67	75.38	62.12

**Table 8:** Comparison with baseline algorithms under SOC and EOC-1.

Method	SOC (%)	EOC-1 (%)
Proposed	99.03	98.08
SVM + PCA	96.52	94.87
SVM + Zernike	95.84	95.14
SVM + EFS	96.02	95.20
SRC	95.64	94.22
A-ConvNet	98.24	96.70
ESENet	98.76	97.23
JSRDeep	98.92	97.64

## Data Availability

The MSTAR dataset is publicly available.
